RETRACTED

# End-of-life discontinuation of destination therapy with cardiac and ventilatory support medical devices: physician-assisted death or allowing the patient to die?

**DOI:** 10.1186/1472-6939-11-15

**Published:** 2010-09-15

**Authors:** Mohamed Y Rady, Joseph L Verheijde

**Affiliations:** 1 Department of Critical Care Medicine, Mayo Clinic Hospital, Mayo Clinic, 5777 East Mayo Boulevard, Phoenix, Arizona, 85054, USA; 2 Center for Biology and Society, School of Life Sciences, Arizona State University, 300 East University Drive, Tempe, Arizona, 85287, USA; 3 Department of Physical Medicine and Rehabilitation, Mayo Clinic Hospital, Mayo Clinic, 5777 East Mayo Boulevard, Phoenix, Arizona, 85054, USA; 4 Department of Biomedical Ethics, College of Medicine, Mayo Clinic, 5777 East Mayo Boulevard, Phoenix, Arizona, 85054, USA

## Abstract

**Background:**

Bioethics and law distinguish between the practices of "physician-assisted death" and "allowing the patient to die."

**Discussion:**

Advances in biotechnology have allowed medical devices to be used as destination therapy that are designed for the permanent support of cardiac function and/or respiration after irreversible loss of these spontaneous vital functions. For permanent support of cardiac function, single ventricle or biventricular mechanical assist devices and total artificial hearts are implanted in the body. Mechanical ventilators extrinsic to the body are used for permanent support of respiration. Clinical studies have shown that destination therapy with ventricular assist devices improves patient survival compared to medical management, but at the cost of a substantial alteration in end-of-life trajectories. The moral and legal assessment of the appropriateness and permissibility of complying with a patient's request to electively discontinue destination therapy in a life-terminating act in non-futile situations has generated controversy. Some argue that complying with this request is ethically justified because patients have the right to request withdrawal of unwanted treatment and be allowed to die of preexisting disease. Other commentators reject the argument that acceding to an elective request for death by discontinuing destination therapy is 'allowing a patient to die' because of serious flaws in interpreting the intention, causation, and moral responsibility of the ensuing death.

**Summary:**

Destination therapy with cardiac and/or ventilatory medical devices replaces native physiological functions and successfully treats a preexisting disease. We posit that discontinuing cardiac and/or ventilatory support at the request of a patient or surrogate can be viewed as allowing the patient to die if--and only if--concurrent lethal pathophysiological conditions are present that are unrelated to those functions already supported by medical devices in destination therapy. In all other cases, compliance with a patient's request constitutes physician-assisted death because of the pathophysiology induced by the turning off of these medical devices, as well as the intention, causation, and moral responsibility of the ensuing death. The distinction between allowing the patient to die and physician-assisted death is pivotal to the moral and legal status of elective requests for death by discontinuing destination cardiac and/or ventilatory medical devices in patients who are not imminently dying. This distinction also represents essential information that must be disclosed to patients and surrogates in advance of consent to this type of therapy.

RETRACTED

## Background

Bioethics and law distinguish between the practices of physician-assisted death and allowing the patient to die, such as by the withdrawal or withholding of life-support treatment in an imminently dying patient. Quill [1] used the term *physician-assisted death *to describe a spectrum of life-terminating medical acts intended to accelerate the dying process and bring about a quick death. Life-terminating acts include voluntary, involuntary, and nonvoluntary active euthanasia, and assisted suicide. Voluntary active euthanasia is the intentional termination of life at the request of the patient or surrogate. Involuntary active euthanasia is the intentional termination of life against the patient's wish. Nonvoluntary active euthanasia is intentionally terminating a patient's life without a request or consent. Prescribing a lethal dose of medication that is ingested by a patient is assisted suicide, whereas giving a lethal dose of a medication to a competent patient who has voluntarily requested to end his or her life constitutes voluntary active euthanasia.

In an acute life-threatening illness or a progressing incurable disease, lethal pathophysiological conditions are set in motion that eventually culminate in death (ie, irreversible cessation of consciousness, respiration, and circulation). In imminently dying patients, these lethal pathophysiological conditions will progress to death despite life-support treatment. Under such circumstances, life-support treatment becomes an impediment to the natural process of dying and physicians withhold and/or withdraw a harmful, ineffective, or burdensome treatment. The term *life-support treatment *is used to mean support of vital functions of respiration and/or circulation in contrast to the term *life-sustaining-treatment*, which includes other treatment avenues such as artificial hydration, nutrition, and hemodialysis. When physicians justifiably withdraw or withhold life-support treatment, they allow patients to die but do not cause, intend, or bear moral responsibility for the patient's death. These medical actions may be perceived as passive euthanasia, but they are not truly euthanasia because there is no intent to terminate life.

RETRACTED

The literature demonstrates that there is little agreement on the meaning of the term "euthanasia" [2]. Introducing adjectives (ie, active, voluntary, involuntary or nonvoluntary) to the word euthanasia only adds confusion to the debate on end-of-life decisions. We agree with the opinion that clearly-defined terms should be used to describe exactly what actions are taking place (eg, withdrawal of treatment, continuation of care, relief of pain, deactivation of medical devices, allowing to die, assisting to die) so as to improve our understanding of what really goes on during end-of-life decisions [2]. The descriptive term of physician-assisted death (dying) is widely used in the medical literature, replacing other emotive terms such as physician-assisted suicide and euthanasia [3-8]. However, the labeling of end-of-life interventions by physicians as either physician-assisted death or palliation is not uniform in similar cases [9]. Differences in the labeling of similar acts performed in end-of-life care can impede societal control even where physician-assisted death has been legalized. Methodological difference in end-of-life interventions such as discontinuing a medical device, administering a specific type or dose of medication, and the time to death may not be helpful in distinguishing acts of palliation from physician-assisted death [10].

Advances in biotechnology have expanded the use of medical devices for permanent mechanical support of respiration and cardiac function in a process known as *destination therapy *when these spontaneous vital functions are irreversibly lost. For example, mechanical ventilators are medical devices used for ventilatory support (VS) of patients with permanent apnea in destination therapy; for the latter purpose, such devices often require a tracheotomy. Single ventricle or biventricular mechanical assist devices and total artificial hearts are medical devices implanted for permanent cardiac support (CS) as destination therapy in patients with end-stage heart failure. We have previously highlighted several ethical challenges in regard to end-of-life care and palliation following destination therapy with the left ventricular assist device (LVAD) [11].

The elective deactivation of mechanical cardiac assist devices has different legal and ethical consequences in non-futile situations compared with futile situations [12]. Physicians often grapple with requests from patients to turn off their LVADs in non-futile situations [13]. In this article, we offer a moral and legal assessment of the decision-making process for discontinuing a constitutive treatment of CS with an LVAD as destination therapy in non-futile situations. We illustrate the similarity to discontinuing, at the patient's request, a constitutive (permanent) treatment of VS with a mechanical ventilator as destination therapy. We argue that compliance with the patient's request to terminate his or her life by discontinuing medical devices for VS or CS is physician-assisted death except under specific circumstances. To distinguish physician-assisted death from allowing a patient to die by deactivation of an LVAD, we evaluate pathophysiological consequences, intention, causation, and moral responsibility for the ensuing death after discontinuation of such a medical device. Responsibility for death is often considered an important factor in the moral distinction between terminating life and letting die [14]. This distinction is not only pivotal to the moral and legal status of requests of discontinuing constitutive VS or CS in patients who are not imminently dying, but it also represents essential information that must be disclosed to patients and surrogates in advance of consent to destination therapy with these medical devices. In assessing the moral and legal status, we differentiate between a constitutive life-support treatment with a medical device as destination therapy and temporary life-support treatment in emergency situations for VS or CS for acute life-threatening illnesses. There is a large body of literature on medical, ethical and legal issues in regard to forgoing temporary or emergent life-support treatment in an acute life-threatening illness. The forgoing of temporary or emergent life-support treatment in an acute life-threatening illness is accepted as morally appropriate, even obligatory, if predicated on true informed consent [15]. In contrast, the literature addressing medical, ethical and legal issues of elective discontinuation of constitutive life-support treatment in non-futile situations is limited and remains controversial [12,14,16-18]. In non-futile situations, the moral significance of acts, omissions and responsibilities in end-of-life interventions continues to be debated in the medical literature [19-21].

RETRACTED

## Discussion

## Hypothetical Scenarios

Consider two hypothetical patients: Adam and David. Adam is a 66-year-old man with traumatic quadriplegia who has been totally dependent on a mechanical ventilator through a tracheotomy because of permanent apnea for two years. David is a 67-year-old man being treated for end-stage heart failure with an LVAD (HeartMate II; Thoratec Corp, Pleasanton, California) implanted two years earlier. Both men live at home with their spouses as their primary caregivers. Adam asks his physician to discontinue VS by turning off the mechanical ventilator and administering medication to ensure a peaceful death. David asks his physician to discontinue CS by deactivating the LVAD and administering medication to induce deep sedation so that he can die a "swift and dignified death." We evaluate whether discontinuing constitutive treatment with VS and CS medical devices, a life-terminating act in these two cases, is either physician-assisted death or death justified by an appeal to the rule of allowing the patient to die. In evaluating both hypothetical scenarios, we focus on the decision and action specifically related to turning off the medical device at the request of the patient. The role of administering medication and pharmacologically inducing deep sedation that results in the deaths of Adam and David will not be discussed. We have argued elsewhere that it is physician-assisted death to administer medication for the purpose of inducing continuous deep sedation to fulfill an elective request for death because of psychological, social, and existential distress [7].

## Types of Treatment With Biotechnological Medical Devices

A treatment is a therapeutic intervention intended to restore body functions and health. Treatment can be temporary (ie, discontinued because of spontaneous recovery of a pathologically disordered body function), or it can be permanent if a specific body function is irreversibly lost. A permanent treatment may be either regulative or constitutive [22]. A regulative treatment attempts to regulate body functions, coaxing the body back toward its own homeostatic equilibrium and baseline health [22]. A regulative treatment is distinct from the organism and extrinsic to its function, whether administered internally or externally to the body. Peritoneal dialysis and hemodialysis are examples of regulative treatment because of the permanent loss of intrinsic kidney function necessary for homeostatic equilibrium [22]. An interruption of regulative treatment results in metabolic derangement but does not generally cause abrupt cessation of vital functions (respiration, circulation, and consciousness) or rapid termination of life.

A constitutive treatment takes over a body function that has been permanently lost and that the body can no longer provide for itself. Although a constitutive treatment is distinct from oneself, it replaces or substitutes for a specific body function essential to life. Mechanical ventilators and cardiac assist devices are biotechnological medical devices that provide VS and CS, respectively. The devices that provide these constitutive treatments are used as destination therapy. They permanently replace vital functions of respiration and circulation that the body can no longer maintain spontaneously. For patients who are totally dependent on a medical device for VS or CS, rapid cessation of vital signs and abrupt termination of life will occur if the operation of the medical device is interrupted. Because of the moral burden of discontinuing a medical device that can result in an abrupt termination of life, criteria have been proposed to differentiate between the two subtypes of constitutive treatment: replacement and substitution [22]. Then, it is claimed that it is morally inappropriate to discontinue a *replacement *treatment because doing so abruptly terminates life and may be viewed as physician-assisted death. In contrast, it is believed to be morally appropriate to discontinue a *substitution *treatment since such an act is simply a matter of allowing the patient to proceed to die. The criteria for categorizing a treatment as a replacement include: 1) its responsiveness to changes in the organism or its environment; 2) properties such as growth and self-repair; 3) independence from external energy sources or supplies; 4) independence from external control by an expert; 5) immunologic compatibility; and 6) physical integration into the patient's body [22].

RETRACTED

The applicability of these criteria in clinical settings appears limited. First, the moral appropriateness or the ethical permissibility of discontinuing constitutive treatment on the premise that it replaces or substitutes for a particular body function is irrelevant regarding end-of-life decisions. There is no absolute standard for judging whether a constitutive treatment with a specific medical device should be considered replacement or substitution of a body function. To morally justify discontinuing these medical devices at the request of patients or surrogates, some physicians consider implantable electronic and mechanical cardiac devices (eg, permanent pacemakers, cardioverter-defibrillators, cardiac resynchronization therapy devices, and ventricular assist devices) as substitution treatment [23,24]. Implantable cardiac devices have also been categorized as life-sustaining treatment to defend the ethical and legal permissibility of device deactivation in patients who are making elective request for death [23]. From a medical perspective, implantable cardiac devices are different from other commonly used life-sustaining treatments, because: (1) these devices can replace native physiological functions of the heart permanently, (2) they control electric and/or mechanical functions of the heart continuously, (3) they are implanted in the body internally, (4) they are responsive to changing body demands intrinsically, and (5) they can induce loss of vital signs rapidly upon deactivation. Deactivating a permanent pacemaker in a pacemaker-dependent patient can induce severe bradycardia or asystole and a rapid cessation of circulation. In a survey of 750 health care providers, 11% of respondents consider that deactivating a permanent pacemaker is euthanasia [25]. In a survey of 185 physicians at a single institution, 9% of physicians characterize the deactivation of a permanent pacemaker in a pacemaker-dependent patient as euthanasia and 19% characterize it as physician-assisted suicide [26]. Deactivating a ventricular assist device can induce a rapid failure or complete arrest of circulation. In a study of end-of-life deactivation of destination LVAD, all patients became unconscious after turning off the device and death followed in < 20 minutes in all cases [27]. The lethal pathophysiology from device deactivation is determined by the type of device and the surgical procedure performed to implant the device in the body and not necessarily by the original pre-existing heart disease (eg. deactivation of a HeartMate II induces an acute aortoventricular regurgitation and deactivating a total artificial heart induces an immediate circulatory arrest). Permanent LVAD support can induce new and irreversible pathological changes in normal heart valves which become the lethal pathophysiology upon device deactivation [28,29].

RETRACTED

A careful assessment of the criteria distinguishing a replacement from a substitution treatment unravels inherent clinical inconsistency and confusion about the classification of implantable mechanical cardiac devices. In destination therapy, the physically implanted LVAD becomes an integral part of the body. It is immunologically compatible with the body and does not require immunosuppressive medications to prevent its biological rejection. LVAD settings are responsive to circulatory demands of the body, but the LVAD lacks the ability to self-repair and depends on an external energy source. Thus, an LVAD might be considered replacement rather than substitution treatment. In contrast, a mechanical ventilator displays few of the criteria of replacement treatment; however, in the scenario of a quadriplegic patient with permanent apnea, many physicians consider a mechanical ventilator replacement rather than substitution treatment. Additionally, one might argue that a transplanted heart is *not *a replacement treatment because of its immunological incompatibility and the requirement for immunosuppressive medications to prevent its biological rejection by the body. Close expert supervision is necessary for monitoring and managing immunosuppressive medications in a transplant recipient. If a recipient refuses to continue on immunosuppressive medications, death ensues because of rejection of the transplanted heart. However, it is argued that a transplanted heart is more likely to be considered replacement rather than substitution of a body function because it cannot be surgically removed without causing a patient's death [22]. The same argument refutes classifying permanent LVAD support as substitution of a body function [24] because the medical device cannot be explanted without causing a patient's death. The arbitrary classification of a constitutive treatment as either replacement or substitution of a body function to ethically permit discontinuation of destination therapy with a medical device in a life-terminating act cannot be substantiated factually but it does give free rein to the construction of what some commentators have referred to as a moral fiction [30].

RETRACTED

Second, irrespective of classifying a constitutive treatment of VS or CS as either a replacement or substitution of body function, circumstantial assessment of the request, causation, intention, and moral responsibility of life termination seriously restricts the ethical permissibility of discontinuing such a treatment. This will be illustrated by the discussion of the hypothetical scenarios of Adam and David below.

Finally, it is important to differentiate the discontinuation of a constitutive treatment in the hypothetical scenarios under discussion from that in the situation where either Adam or David would be imminently dying from a lethal pathophysiological condition independent of vital body functions (ie, ventilatory and cardiac functions) supported by respective medical devices. Examples of life-ending pathophysiological conditions, irrespective of continued VS or CS by medical devices used in destination therapy, may include the irreversible loss of consciousness from a catastrophic neurological event, peripheral vascular collapse and shock from an overwhelming infection, and refractory hypoxia from worsening lung disease or disseminated malignancy. Could this difference mark a legally clear and clinically relevant distinction between physician-assisted death and allowing patients to die?

## Moral Fiction About Discontinuing Constitutive Medical Devices

Moral fictions are false beliefs upholding entrenched moral positions in the face of a conduct or practice in tension with established moral norms [30]. Moral fictions can be culturally entrenched, even when their falsity is exposed. Moral fictions are created from flawed interpretations of facts or false assumptions about a certain medical practice. When a specific medical practice, viewed candidly, appears to conflict with established moral norms, there is a strong incentive to construe this practice in a way that seems to remove the moral conflict. Moral fictions counteract a cognitive dissonance originating from an inconsistency between the facts about that medical practice and the prevailing moral norms. For critics who recognize the cognitive dissonance, moral fictions appear to be patently false [30].

RETRACTED

When the discontinuation of destination therapy with a medical device for VS or CS results in a life-terminating act, moral fiction is often invoked to avoid construing such an act as physician-assisted death. Classifying a constitutive treatment as a substitution instead of the replacement of a body function, and then conveniently assigning an ethical permissibility to discontinuing the former but not the latter is illustrative of a moral fiction. Moral fictions are intended to convert an ethically challenging life-terminating act, whether inducing deep coma with medication and/or discontinuing constitutive VS or CS at the request of a patient or surrogate, into an act that appears congruent with the prevailing moral norm; that is physicians must not kill or assist in killing patients.

The pathophysiological conditions leading to death can distinguish allowing a patient to die from physician-assisted death. Allowing a patient to die is withholding and/or withdrawing life-support treatment for a lethal pathophysiological condition set in motion by a newly developed acute life-threatening illness or by a chronic treatment-refractory advanced disease. Physician-assisted death is creating a new, nontherapeutic, lethal pathophysiological condition in a human being with the intention of thereby causing or hastening that person's death [22]. Can this pathophysiological differentiation adequately categorize a physician's action of discontinuing medical devices for VS or CS?

It is difficult to contend that, in destination therapy, a medical device for VS or CS that replaces basic vital body functions is extrinsic to or separate from the patient's identity. When a mechanical cardiac assist device such as an LVAD is successfully implanted, the recipient perceives this device as part of his or her body image and sense of self [31]. A patient living with an LVAD develops an identity that is physically, emotionally, and psychologically dependent on the implanted device [32-34]. Additionally, a patient with a total artificial heart has no native cardiac function because the left and right ventricles are surgically removed to implant the medical device. A patient's circulation is then totally dependent on normal operation of the medical device. This is not different from a patient's respiration that is totally dependent on normal operation of the mechanical ventilator because of permanent apnea. The medical device becomes a replacement for that body function which is essential for life and thus is an integral part of the restored physiology of the patient. The medical device and its constitutive function are part of the integrated unity of the patient as an intact, living, individual organism. In destination therapy, medical devices permanently replace VS and CS and constitute the vital signs of respiration and circulation for that patient, respectively. From a pathophysiological perspective, turning off a mechanical ventilator or an LVAD creates a new and nontherapeutic lethal pathophysiological condition by interrupting the patient's vital signs and resulting in death through cessation of circulation, respiration, and consciousness. To discontinue such treatment not only discontinues the treatment of preexisting disease but also introduces new and nontherapeutic lethal pathophysiological conditions in the patient. The medical device has successfully treated the underlying preexisting disease (some patients may even mistakenly view it as a cure), which is also the original intent of consent for destination therapy with a medical device. In the absence of a newly developed acute life-threatening illness that sets in motion a lethal pathophysiological condition regardless of VS or CS, turning off a mechanical ventilator or an LVAD would appear to result in a rapid cessation of vital functions, thus leading to death. When regulative and constitutive destination medical devices are discontinued the ensuing lethal pathophysiological conditions can be different. Discontinuing a regulative treatment (eg, hemodialysis) does not generally result in an abrupt interruption of vital signs but, instead, causes a gradual lethal metabolic disorder. Upon discontinuing both regulative and constitutive destination medical devices, new nontherapeutic lethal pathophysiological conditions are set in motion causing death, but with different end-of-life trajectories.

RETRACTED

The objective assessment of a patient's request, causation, intention, and moral responsibility reveal two additional moral fictions pertaining to the argument that turning off the medical devices in the hypothetical scenario of Adam and David would not be physician-assisted death. The first moral fiction concerns 1) the nature of the patient's request; 2) the nature of the act that the physician is asked to perform in either case; 3) the causal relationship between the act of treatment withdrawal and the patient's death; and 4) the intention of the physician who accedes to such a request. The second moral fiction is related to erroneous judgments about moral responsibility that are based on these mistaken factual claims. When shorn of these moral fictions, compliance with the request of either Adam or David would more appropriately be defined as physician-assisted death.

## Request and Consent for Discontinuing Constitutive Medical Devices

Respect for autonomy and self-determination entails the right of a competent patient to accept or refuse a particular treatment at a specific time. Rescinding a prior "informed" consent to a constitutive treatment or destination therapy with a medical device might be considered to be supported by the patient's right to self-determination. If so, Adam and David would be exercising their rights of autonomy and self-determination when they refuse continued constitutive treatment with a medical device. Bioethicists often argue that withdrawing any life-support treatment is morally and legally similar to withholding life-support treatment in the context of fatal disease at the end of life. The question then becomes whether this ethical argument can be applied to a constitutive treatment with a medical device that is *successfully *treating a patient's *fatal *disease without the presence of any new lethal pathophysiological condition. Can this ethical argument uphold the notion that Adam's and David's requests are simply a matter of allowing patients to die rather than a case of physician-assisted suicide or physician-assisted death?

The term *suicide*, from the Latin words *sui caedere*, means the intentional killing of oneself. Both Adam and David are making suicidal requests because they believe that depending on artificial machines for basic vital functions has made life too burdensome. Although the concept of rational suicide seems nonsensical to those who believe that it is always irrational to opt for death, the definition of suicide in these two hypothetical cases might also be rejected because neither patient is physically capable of causing his own death. Both must seek a physician's assistance to do so. Both want to die because they believe that only death will free them from an increasingly intolerable condition; thus, it is their requests for assistance in dying that set in motion the causal chain leading to death if their physicians comply with those requests. Logically, however, we might infer that both patients are requesting assisted suicide because they need the help of someone else to actualize their wish to die. Regardless of the suicidal nature of such a request, one could argue that a physician who accedes to it is not engaging in assisted suicide because the immediate death-causing act is performed by the physician rather than the patient. In true assisted suicide, the act causing immediate or imminent death is performed by the patient. Physically capable patients can also disconnect themselves from either mechanical ventilators or LVADs and intentionally cause their own death. But as mentioned previously, the two ethical arguments (ie, self-determination and moral equivalency of withholding or withdrawing treatment) may seem to support the notion that discontinuing medical devices in both cases is simply a matter of allowing the patient to die. However, the assertion that the requests of Adam and David do not involve suicide is grounded in a moral fiction. There is no basis for not describing such life-terminating acts as physician-assisted death. Despite the unequivocal consequence of fulfilling such a request, some physicians might reject the label of assisted death when they comply with it because of the moral fictions regarding causation and intention.

RETRACTED

### Causation

In these two hypothetical scenarios, both Adam and David have the potential to live for an unknown time--even years--supported by their respective medical devices: a ventilator and an LVAD. What explains Adam's death after withdrawal of VS is not the course of his spinal cord injury but the very act of turning off the ventilator. David's death after withdrawal of CS is not caused by the natural progression of his heart disease, which is being successfully treated by an LVAD, but rather by the act of deactivating the LVAD. Turning off the ventilator or deactivating the LVAD is thus the proximate and immediate cause of death. This conclusion is supported by the proposed pathophysiological differentiation between allowing the patient to die and physician-assisted death. In addition, disconnecting the ventilator or deactivating the LVAD without the patient's consent would constitute an act of nonvoluntary active euthanasia.

The withdrawal of a constitutive VS or CS, when followed immediately by death, is a life-terminating intervention. Indeed, the very fact that a mechanical ventilator can sustain life for patients incapable of spontaneous breathing implies that stopping mechanical ventilation will end life. Similarly, the very fact that a mechanical cardiac assist device can sustain life for patients incapable of spontaneous circulation signifies that stopping such a device will end life. In other words, the power to sustain life by technological means goes hand in hand with the power to end life when those means are withdrawn.

RETRACTED

The discontinuation of the ventilator in Adam's case or the deactivation of the LVAD in David's case is what results in dying at the time and in the manner each has chosen for ending his life. They may opt for an elective request to end life because of the belief that suffering is pointless, the fear about future suffering or dependency, tiredness with living, loss of dignity, the wish to die with dignity, a desire to determine the time of death, a desire to avoid being an economic burden on others, concern about family fatigue, or intolerable psychological or social suffering for themselves or their families. These reasons are similar to those of patients requesting physician-assisted death [35]. Hence, we conclude that the causation argument in describing either Adam's death after turning off the ventilator or David's death after deactivating the LVAD as merely allowing death rather than directly causing death can only be made on the basis of moral fiction.

### Intention

Withdrawing a life-support treatment is considered legally and ethically permissible when it is based on the valid refusal of treatment by a competent patient or an authorized surrogate decision-maker because of the prior preferences of the patient or the sound judgment of the surrogate about the patient's best interests [15]. These end-of-life decisions are made everyday for critically ill patients with acute life-threatening and nonsurvivable illnesses who are on life-support treatment in an intensive care unit. For an imminently dying patient who is likely to die regardless of life-support treatment, the intention to discontinue that treatment is to remove an impediment to a natural death.

Physicians who view the plans of Adam and David as reasonable given their circumstances, values, and preferences, and who may be prepared to assist with the execution of those plans, intend not only to respect the autonomous choices of the patient but also to cause the patient's death. A survey of end-of-life decisions in 6 European countries (Belgium, Denmark, Italy, the Netherlands, Sweden, and Switzerland) demonstrates that almost half of the physicians reported an explicit intention to hasten death when they elected to withdraw life-support treatment [36]. In a survey of intensive care units in 17 European countries, Sprung et al reported a similar gray area in end-of-life interventions between acts to relieve pain and suffering and acts intended to shorten or hasten the dying process [37]. Neither the type and dose of medication nor the time to death could discriminate between acts intended to palliate symptoms from acts intended to hasten the dying process upon withdrawal of life support. Physicians' true intentions are private and often undisclosed in end-of-life care [38]. Intending to hasten death is the same as intending to cause death because hastening death causes death to occur earlier than it otherwise would.

RETRACTED

### Moral Responsibility

Once we uncover the moral fictions concerning the causation and intention about discontinuing destination therapy with VS and CS medical devices in the cases of Adam and David, it becomes clear that denying the moral responsibility of the physician for his or her role in their deaths is part of those fictions (Table 1). Specifically, a physician is morally responsible for causing a patient's death either by turning off a ventilator or by deactivating an LVAD when this life-terminating act can be attributed to the physician from a moral perspective. Is causing death something that the physician did voluntarily and knowingly, so that it can be attributed to him? Physicians are morally responsible for what they intend to do, as well as for what they do knowingly or negligently.

**Table 1:** End-of-Life Discontinuation of Constitutive Medical Devices for Ventilatory and Cardiac Support in Destination Therapy

Consideration	Hypothetical Scenario	
	**Discontinuation of Constitutive Ventilatory Support With MV (Adam**^**a**^**)**	Discontinuation of Constitutive Cardiac Support With LVAD **(David**^**b**^**)**
**Pathophysiology**		

Introducing new, nontherapeutic, lethal conditions	Yes	Yes

**Request/Consent**		

Is it suicide?	Yes	Yes

Is it assisted suicide?	Yes	Yes

**Causation**		

Is the physician causing death?	Yes	Yes

Is it an active intervention?	Yes	Yes

**Intention**		

Is the physician intending death?	Sometimes Yes, sometimes No	Sometimes Yes, sometimes No

**Moral Responsibility**		

Is the physician morally responsible for death?	Yes	Yes

Is it physician-assisted death?	Yes	Yes

Abbreviations: LVAD, left ventricular assist device; MV, mechanical ventilator.

^a^Adam is a quadriplegic patient on permanent ventilatory support with a mechanical ventilator (MV) for two years. Adam asks his physician to administer medication to induce deep sedation and to turn off the MV so that he can die peacefully.

^b^David is a patient with end-stage heart failure who has had permanent implantation of a HeartMate II (Thoratec Corp, Pleasanton, California) left ventricular assist device (LVAD) as destination therapy two years earlier. David asks his physician to administer medication to induce deep sedation and to deactivate the LVAD so that he can die quickly and with dignity.

RETRACTED

The moral responsibility of assisting in a life-terminating act by discontinuing a destination therapy with a medical device is not lessened by the consent of a competent patient or a legally authorized surrogate decision-maker. The moral responsibility for causing death is shared by the patient or surrogate and the physician. The primary responsibility rests with the patient or surrogate, but prior authorization for treatment withdrawal does not negate the physician's role and moral responsibility for discontinuing a constitutive VS or CS device and thus for causing the ensuing death (Figure 1).

**Figure 1:** **End-of-Life Discontinuation of Destination Therapy with Ventilatory and Cardiac Support Medical Devices**. Mechanical ventilators and cardiac assist devices can replace native vital functions of respiration and circulation in destination therapy, respectively. Respiration and circulation become totally dependent on normal operation of these medical devices. Discontinuing mechanical ventilators and cardiac assist devices used as destination therapy can create nontherapeutic and lethal pathophysiological conditions and become the life-terminating events. The absence of concurrent lethal pathophysiological conditions that are set in motion by a newly developed acute life-threatening illness and/or a terminal disease, unrelated to the body function supported by these medical devices, refutes the notion that discontinuing destination therapy at the patient's or surrogate's elective request for death is simply allowing the patient to die. Assessment of intent, causation, and moral responsibility of the ensuing death upon discontinuing the medical device is consistent with physician-assisted death. Discontinuing permanent mechanical ventilators and cardiac assist devices can be viewed as allowing the patient to die if--and only if--concurrent lethal pathophysiological conditions are present that are unrelated to vital functions already supported by these medical devices. Examples of concurrent lethal pathophysiological conditions from an acute life-threatening illness and/or a chronic treatment-refractory advanced disease may include: irreversible loss of consciousness from a catastrophic neurological event, peripheral vascular collapse and shock from an overwhelming infection, multiple organ failures, refractory hypoxia from worsening lung disease or disseminated malignancy.

## Moral Assessment of Discontinuing Constitutive Medical Devices

Finally, we come to the differential moral evaluation of physician-assisted death versus allowing the patient to die in response to the patient's request or the patient's refusal of continued treatment by a ventilator or an LVAD. Per the premise of self-determination, patients have both a moral and a legal claim-right to stop unwanted treatment, which physicians and health care institutions are obligated to respect. The US courts have ruled that the right to make decisions about medical treatment is both a common law right based on bodily integrity and self-determination, as well as a constitutional right based on privacy and liberty. Some commentators interpret the court ruling to uphold the patient's right to refuse an ongoing treatment or a successful destination therapy with a permanent medical device implanted in the body [23,24]. On this premise, deactivation of a permanent medical device in a life-terminating act, upon an elective request for death, is considered a patient's right. Compliance with the request, as a respect for this right, is regarded as allowing the patient to die and not assisting in death even though the patient is neither terminally ill nor imminently dying [23]. The validity of this right is not contingent on the physician's endorsement of the patient's reasons for treatment refusal. Does the right to refuse a treatment imply the right to demand a life-terminating act? The right to refuse a treatment, however, is not the same as the right to receive any treatment insisted upon by the patient or a surrogate. Therefore, it can be argued that a patient's right to receive or demand a lethal treatment or intervention (eg, deactivating a medical device) is open to questioning. Although patients arguably have a moral liberty-right of noninterference by others when requesting an abortion or assisted-death, they do not have a claim-right to receive an abortion or assisted-death upon demand if the physician is unwilling to provide such a service. Can a patient's autonomy legitimize a physician's role in assisted death? In *Vacco v. Quill*, the US Supreme Court "...distinguished between the refusal of lifesaving treatment and assisted suicide [assisted death], by noting that the latter involves the criminal elements of causation and intent. No matter how noble a physician's motives may be, he may not deliberately cause, hasten, or aid a patient's death [39]." In *Washington v. Glucksberg*, "the Court held that the right to assisted suicide [assisted death] is not a fundamental liberty interest protected by Due Process Clause [of the Fourteenth Amendment of the US Constitution] since its practice has been, and continues to be, offensive to our national traditions and practices. Moreover, employing a rationality test, the Court held that... [state's] ban was rationally related to the state's legitimate interest in protecting medical ethics, shielding disabled and terminally ill people from prejudice which might encourage them to end their lives, and, above all, the preservation of human life [40]."

RETRACTED

Allowing a patient to die by an act of omission (eg, withholding a treatment) may have different psychological effects on healthcare providers than allowing a patient to die by an act of commission (eg, turning off a medical device). Furthermore, turning off a VS or CS medical device because of a rapidly progressing fatal illness from which death is imminent may be psychologically different from a situation lacking such an illness. For example, if Adam were to develop a life-threatening kidney infection with septic shock resulting in multiple organ failure, then continuing VS would be unlikely to prevent him from dying. In that scenario, turning off the ventilator is unlikely to be the proximate cause of Adam's death. Likewise, if David were to suffer a catastrophic, bilateral cerebral hemorrhage resulting in an irreversible coma, then he would be unlikely to survive despite continued CS. In such a case, deactivating the LVAD is unlikely to be the proximate cause of death. The psychological challenges of complying with such requests to discontinue the medical device are amplified because they do not differ in intention, causation, and moral responsibility from those inherent in physician-assisted death. Administering lethal doses of medication (an ordinary tool of medicine) to cause a patient's death is active euthanasia. Discontinuing a constitutive VS or CS (ie, turning off a technology tool of medicine) results in death. In both situations, there are no real or meaningful differences in the physician's role. In both cases, the patients are seeking a swift death with physician assistance and there is no relevant difference in the causation and moral responsibility for their deaths.

## The Moral Reality of Life-terminating Medical Decisions

The moral norm in the practice of medicine is that physicians must not kill patients or intend their deaths. With few exceptions, such as capital punishment and just war, US law treats the intentional causing of death as criminal homicide. In order for the practice of discontinuing a constitutive treatment of VS or CS to be permitted legally and ethically, moral fictions about life-terminating decisions (in terms of intention, causation, and responsibility) must be accepted as valid justifications. One can choose to perceive the discontinuation of VS or CS as no different from its withdrawal in imminently dying patients, *as if *it is not suicide or assisted suicide, *as if *it is passive euthanasia and merely allowing death, and *as if *death is not necessarily intended. Consequently, when discontinuing a constitutive treatment of VS or CS, physicians would not be considered legally responsible for causing the death of their patients and not be guilty of homicide. Perhaps more importantly, upholding such a perception permits patients and families who are morally opposed to suicide to accept the life-terminating decision to discontinue VS or CS medical devices being used for destination therapy.

RETRACTED

Uncovering the plain empirical fact that discontinuing a destination therapy is, in essence, physician-assisted death might also have unintended consequences on medical practice. Physicians may become reluctant to engage patients and family members in conversations about end-of-life care and the anticipated need for discontinuing such devices. Physicians may become resistant to requests from patients or families to discontinue such medical devices in clinical situations when death is imminent from lethal pathophysiological conditions developing from new life-threatening illnesses. Moral and public acceptance of VS and CS medical devices as destination therapies might be imperiled. Recognizing the moral predicament of discontinuing a constitutive treatment might contribute to unease or reluctance on the part of patients and families to consent to destination therapy with medical devices. In addition, the resulting reluctance and declining use of destination therapy with VS and CS medical devices could have negative financial consequences on medical device manufacturers and institutions that provide such specialized services.

The inherent growing pressure within the medical community to expand life-prolonging medical technology introduces the risk of abandonment of one of the most important ethical norms in the practice of medicine: physicians must not harm or kill their patients. Discontinuing certain types of life-sustaining technology [41,42] and medical devices [23] (eg, deactivation of antibradycardia pacing in a pacemaker-dependent patient) in a life-terminating act is prohibited by law in some countries. Some US states have enacted a Death with Dignity Act to alleviate the tension between traditional norms of medical practice and the reality of intentional life-terminating acts by physicians [7]. However, legalizing physician-assisted death may not be the best resolution of this moral conflict. Legalization of physician-assisted death in medical practice can lead to the potential abuse of voluntary active euthanasia because any person can be killed by lethal injection, whereas withdrawing life-support treatment can kill only those who are on life support and require it to continue living. Legalization of physician-assisted death might also expand the withdrawal of life-support treatment with no consent in incompetent and vulnerable patients. Life-ending interventions without explicit consent are already being performed on patients whose diseases have unpredictable end-of-life trajectories [8].

RETRACTED

It is difficult to continue to pass off a moral fiction as the truth once the fiction has been exposed. However, indulging in moral fictions may have worse consequences than facing the moral truth and dealing with the conflict about certain life-terminating medical practices. By failing to unravel and abandon moral fictions, we risk perpetuating an unregulated practice that sends the medical profession and society down a slippery slope distant to the fundamental moral values of humanity. Facing the moral truth is essential to preserving society's trust in the integrity of the medical profession and its practice. Confronting the moral truth should be a powerful motive to explore ways of resolving conflict between certain prevailing practices and the moral norms of the medical profession.

## Summary

Advances in biotechnology medical devices have produced constitutive (permanent) treatment with mechanical ventilators and cardiac assist devices for VS and CS as destination therapy. The moral and legal assessment of the appropriateness and permissibility of complying with a patient's requests to electively discontinue destination therapy in a life-terminating act in non-futile situations continues to generate controversy. Some argue that complying with this request would be ethically justified because patients have the right to request withdrawal of unwanted treatment and be allowed to die of preexisting disease. Destination therapy with VS or CS should be considered a successful treatment of the original preexisting disease. Discontinuing VS or CS at the request of the patient or surrogate can be viewed as allowing to die, if--and only if--concurrent lethal pathophysiological conditions are present that are unrelated to the functions already supported by the medical devices in destination therapy. In all other cases, acceding with a patient's request constitutes physician-assisted death because of the pathophysiology induced by the turning off of these medical devices, as well as the intention, causation, and moral responsibility of the ensuing death. The distinction between allowing the patient to die and physician-assisted death is not only pivotal to the moral and legal status of elective requests for death by discontinuing destination cardiac and/or ventilatory medical devices in patients who are not imminently dying, but it also represents essential information that must be disclosed to patients and surrogates in advance of consent to this type of therapy.

RETRACTED

## Abbreviations

CS: cardiac support; LVAD: left ventricular assist device; VS: ventilatory support

## Competing interests

The authors have no affiliation or financial involvement to disclose with any organization or entity with a direct financial interest in the subject matter or materials discussed in the manuscript. The authors declare that they have no competing interests.

## Authors' contributions

MYR and JLV attest that they have made substantial contributions in drafting the manuscript and revising it critically for important intellectual content, that they have given final approval of the version to be published, and that they have participated sufficiently in the work to take public responsibility for appropriate portions of the content. Both MYR and JLV have read and approved the final manuscript.

## Pre-publication history

The pre-publication history for this paper can be accessed here:

http://www.biomedcentral.com/1472-6939/11/15/prepub
